The article "Artificial Intelligence Algorithm with ICD Coding Technology Guided by the Embedded Electronic Medical Record System in Medical Record Information Management" was published in 2021. Journal: J Healthc Eng.

# Artificial Intelligence Algorithm with ICD Coding Technology Guided by the Embedded Electronic Medical Record System in Medical Record Information Management

**DOI:** 10.1155/2021/3293457

**Published:** 2021-08-30

**Authors:** Cheng Wang, Chenlong Yao, Pengfei Chen, Jiamin Shi, Zhe Gu, Zheying Zhou

**Affiliations:** ^1^Medical History Room, Shanghai First Maternity and Infant Hospital, Shanghai 200000, China; ^2^Department of Information, Children's Hospital Affiliated to Jiaotong University, Shanghai 200000, China; ^3^Unionnet Co. Ltd., Shanghai 200000, China

## Abstract

The study aims to explore the application of international classification of diseases (ICD) coding technology and embedded electronic medical record (EMR) system. The study established an EMR information knowledge system and collected the data of patient medical records and disease diagnostic codes on the front pages of 8 clinical departments of endocrinology, oncology, obstetrics and gynecology, ophthalmology, orthopedics, neurosurgery, and cardiovascular medicine for statistical analysis. Natural language processing-bidirectional recurrent neural network (NLP-BIRNN) algorithm was used to optimize medical records. The results showed that the coder was not clear about the basic rules of main diagnosis selection and the classification of disease coding and did not code according to the main diagnosis principles. The disease was not coded according to different conditions or specific classification, the code of postoperative complications was inaccurate, the disease diagnosis was incomplete, and the code selection was too general. The solutions adopted were as follows: communication and knowledge training should be strengthened for coders and medical personnel. BIRNN was compared with the convolutional neural network (CNN) and recurrent neural network (RNN) in accuracy, symptom accuracy, and symptom recall, and it suggested that the proposed BIRNN has higher value. Pathological language reading under artificial intelligence algorithm provides some convenience for disease diagnosis and treatment.

## 1. Introduction

With the improvement of living standards, people's attention to their health is also increasing. At the same time, they are concerned about the medical conditions and facilities of the hospital. The hospital will conduct statistical analysis and comparison of the annual medical data to form an indicator of medical quality management [1]. Most of the data in the medical industry come from electronic medical records (EMRs). EMR is also called computerized medical record system or computer-based patient record (CPR). It is a digital medical record saved, managed, transmitted, and reproduced by electronic devices (computers, health cards, etc.) to replace handwritten paper medical records. Its content includes all the information of paper medical records. The National Institute of Medicine defines EMR as an electronic patient record based on a specific system, which provides users with the ability to access complete and accurate data, warnings, prompts, and clinical decision support systems.

Through the extraction and statistical analysis of these data, relevant indicators are formed to provide convenience for medical personnel, which help them better understand the relevant medical conditions and improve the quality of medical care [2]. With the rise and wide application of computer network technology, its application in the medical industry is becoming more common. Most medical institutions use a unified medical record front page, which provides great convenience for the information statistics of the medical industry [3]. The medical record records the detailed condition of the patient, from the initial diagnosis to the final treatment result, which provides a detailed basis for the follow-up [4, 5]. The detailed record of the patient's condition in the medical record provides important support for medical staff to understand the patient's condition. Both the past medical history and the current diagnosis and treatment of diseases can be consulted [6]. With the development of electronic information on the Internet, case records have also changed from the original paper version to an electronic version, completing the digital management mode of medical records [7, 8]. Electronic cases have greatly improved the efficiency of using medical records. The use of EMRs provides convenience for medical staff and management staff.

ICD coding technology is a relatively complete and mature disease-coding method. Almost every hospital unit uses its rules to code diseases on the front page of medical records [9]. The combination of English and numbers is used for coding to avoid coding inconsistencies [10]. It promotes exchanges between people from different countries and regions. With the continuous improvement of disease classification by scholars, more and more disease types are covered [11]. The coding method is characterized by scientificity, integrity, applicability, and operability. Therefore, it is widely used in the field of medicine [12]. In clinical medicine, the use of LCD can bring great convenience, unify the code for global diseases, facilitate researchers' research, and contribute to the development of medicine.

In this experiment, the statistical analysis of the first page of medical records is conducted through the sample survey. The causes of errors in the disease classification on the first page of the medical record are analyzed and summarized. Meanwhile, the embedded medical record information knowledge system is established, and the NLP-BIRNN algorithm is used to optimize the medical record text. Also, the detailed improvement measures are proposed to provide a basis for the investigation of disease classification.

## 2. Materials and Methods

### 2.1. Experimental Materials

The data were randomly selected from the EMR database of our hospital, and the patient medical records and disease diagnostic code data on the front pages of 8 clinical departments of endocrinology, oncology, obstetrics and gynecology, ophthalmology, orthopedics, neurosurgery, and cardiovascular medicine were collected.

### 2.2. Case Statistics

The medical record information is randomly extracted from the EMR management system for analysis. Statistics on the diagnosis selection and the number of disease-coding errors are conducted. The statistical analysis of the data of clinicians and medical coders before and after training is performed. Through research, self-examination, training, and feedback, the disease-coding knowledge topics of the above eight clinical departments are explored. The coder calls up the medical record data of a certain department. According to ICD-10's undergraduate disease-coding rules, such as clinical knowledge and main diagnosis selection principles of the disease's physiological mechanism, development process, clinical manifestations, and treatment methods, the disease-coding process is conducted. During the coding process, the coder must carefully read the case, especially the admission records (judgment of the main diagnosis selection), surgical records (surgical name, postoperative method, surgical grade, surgical incision, and anesthesia method), course records (development of the disease, such as whether the disease is aggravated, whether it is improved, and whether it is treated), and discharge records (diagnosis and treatment process, whether the diagnosis at admission and discharge are consistent). Pathology, imaging, ultrasound, and laboratory reports should also be paid attention to.

### 2.3. Self-Examination and Training

According to the results, the coder reexamines the previous medical records, mainly checking the diagnosis selection and disease coding. Statistics on the data of diagnosis selection errors and disease-coding errors are conducted. Then, ICD-10 training will be given to the relevant doctors and coders of the above eight clinical departments on the problems examined this time.

### 2.4. Feedback

The coder compares and analyzes the data of main diagnosis selection errors and disease-coding errors before and after the training. The results are then shared to the relevant personnel with feedback, to explore rectification measures and improve the coding level.

### 2.5. Establishment of Embedded EMR Information Knowledge System

The system establishes conditions. First, conditions are written based on the writing standard of medical records stipulated by the national health department. The data content expressed in the medical record should be a common medical term without ambiguity. Second, the knowledge system must contain descriptive and conclusive knowledge about medical records. Descriptive knowledge refers to the detailed description of the disease. For example, the types of cold are wind chill and wind heat and their common symptoms are headache and cough, which is descriptive knowledge. On the contrary, it is conclusive knowledge to judge the type of cold according to the description of the disease. The knowledge system needs to combine the structured input interface of medical records and provide a selective input prompt based on the user input. Third, the medical record information is stored as an XML document, which has hierarchical structure. The knowledge base is also represented by the hierarchical XML document to achieve efficient synchronization of medical record input interface, which corresponds to the medical record information document. For some simple information input without prompt, the node can be set to null value. For items with multiple choices, multiple child nodes can be set when prompted, read into memory, and displayed in the medical record interface for users to choose. Fourth, the semantics should be concise and include the hints about limiting the use of characters.

The information base of the embedded medical record knowledge system contains knowledge, as shown in Table 1:

There are seven pages in the embedded EMR input system, and seven XML documents of medical record knowledge base are established accordingly. When doctors create a new medical record page, the system will automatically call the knowledge base XML document according to the current page. When doctors input specific document node information, they can input medical record information according to prompt operation to improve the recording speed and reduce expression errors.

### 2.6. Steps of NLP-BIRNN Algorithm

First, the data preprocessing of EMR is carried out, including data processing, cleaning, and screening.

Second, NLP based on medical tagging (medical record tagging, character extraction, word vector transformation, deep neural network, automatic tagging, and feature vector splicing) and NLP without medical tagging (no medical record, part of speech tagging, keyword selection, word vector transformation, and feature vector splicing) are performed.

Third, calculation is done. The symptom feature vectors involved in NLP solutions are normalized, and the values at each position of vector data are limited to [0, 1]. The ICD is coded by one hot representation to become the tag of deep learning training. The normalized feature vector and label are imported into the deep learning model for training, the auxiliary diagnosis model is obtained, and the test set is used to complete the test of the model results.

### 2.7. Data Analysis

The SPSS24.0 software was adopted for data statistics and analysis. The difference between the two groups of data was analyzed by the *t*-test. The count data were compared by the Chi-square test. *P* < 0.05 indicated significant difference, and *P* < 0.01 indicated highly significant difference.

## 3. Results

### 3.1. CT and Ultrasound Images of Some Diseases

At present, the diagnosis basis of 2019 novel coronavirus (2019-nCoV) is mainly nucleic acid testing and medical imaging detection. The combination of the two is more conducive to diagnosis. It is found from the announcement of officially confirmed cases that some patients showed a positive result after more than 2 nucleic acid tests and even showed a positive result after the fifth nucleic acid test. Therefore, while performing nucleic acid testing, lung CT imaging examination is carried out. Patients with lung CT presenting with signs of acute inflammation should be admitted as soon as possible in accordance with the principle of “suspected disease is always present.” The CT and ultrasound results of some diseases are shown in Figure 1.  Figure 1(a) is a chest CT image of coronavirus disease 2019 (COVID-19).  Figure 1(b) is a segmented image of the pneumonia-infected area.  Figure 1(c) is a CT of the abdomen. The accuracy of diagnosing the mild fatty liver using CT is 88.75%.  Figure 1(d) is an ultrasound image of the abdomen. The accuracy of diagnosing the mild fatty liver using ultrasound is 73.75%. It shows that CT diagnosis is more accurate than ultrasound diagnosis.

### 3.2. Results of Main Diagnosis Selection Errors and Disease-Coding Errors of the Obstetrics and Gynecology Department

Results of main diagnosis selection errors and disease-coding errors of the obstetrics and gynecology department are shown in Figure 2.  Figure 2(a) is the results of the main diagnosis selection errors. There are 280 errors in the discharge case statistics before the training and 80 errors after the training. The statistics on the four types of main diagnosis selection errors are conducted, including that C-section is the main diagnosis, singleton live birth diagnosis is the first, tumor morphological coding is the main diagnosis, and major treatable diseases are not major diagnosed. It is found that the difference in each index between groups before and after training is significant (*P* < 0.05).  Figure 2(b) is the results of disease-coding errors. There are 240 errors in the discharge case statistics before the training and 60 errors after the training. The statistics on the four types of disease-coding errors of pregnancy hypertension, premature rupture of membranes, tumors, and mass, and vomitus gravidarum are conducted. It is found that the difference in each index between groups before and after training is significant (*P* < 0.05).

### 3.3. Results of Main Diagnosis Selection Errors and Disease-Coding Errors of the Endocrinology Department

Results of the main diagnosis selection errors and disease-coding errors of the endocrinology department are shown in Figure 3.  Figure 3(a) is the results of the main diagnosis selection errors. There are 180 errors in the discharge case statistics before the training and 50 errors after the training. The statistics on the three types of main diagnosis selection errors are conducted, including that the treatment of the disease is not a major diagnosis, multiple complications are not primarily diagnosed, and no major diagnosis is made for a single complication. It is found that the difference in each index between groups before and after training is significant (*P* < 0.05).  Figure 3(b) is the results of disease-coding errors. There are 160 errors in the discharge case statistics before the training and 30 errors after the training. The statistics on the five types of disease-coding errors are conducted, including the merge coding error, no additional coding used, neonatal diabetes mellitus, gestational diabetes mellitus, and screening for diabetes. It is found that the difference in each index between groups before and after training is significant (*P* < 0.05).

### 3.4. Results of Main Diagnosis Selection Errors and Disease-Coding Errors of the Orthopedics Department

Results of the main diagnosis selection errors and disease-coding errors of the orthopedics department are shown in Figure 4.  Figure 4(a) is the results of the main diagnosis selection errors. There are 120 errors in the discharge case statistics before the training and 30 errors after the training. The statistics on the four types of main diagnosis selection errors are conducted, including that the removal of the immobilization device does not make the primary diagnosis, multiple site fractures are not primarily diagnosed, the main diagnosis is made for the cause of injury, and postoperative complications of fractures are not primarily diagnosed. It is found that the difference in each index between groups before and after training is significant (*P* < 0.05).  Figure 4(b) is the results of disease-coding errors. There are 160 errors in the discharge case statistics before the training and 25 errors after the training. The statistics on the four types of disease-coding errors are conducted, including that the coding of damage sites is inaccurate, the postoperative complication coding is not accurate, the main treatment is uncoded, and the cause of injury poisoning is not clear. It is found that the difference in each index between groups before and after training is significant (*P* < 0.05).

### 3.5. Results of Main Diagnosis Selection Errors of the Oncology and Neurosurgery Department

Results of the main diagnosis selection errors of the oncology and neurosurgery department are shown in Figure 5.  Figure 5(a) is the results of the main diagnosis selection errors of oncology. There are 260 errors in the discharge case statistics before the training and 60 errors after the training. The statistics on the four types of main diagnosis selection errors are conducted, including that the primary diagnosis of the tumor is not made in Z code, using Z code to make the primary diagnosis is inaccurate, major diagnosis is not made for the major treatment of disease, and tumor morphology code is the main diagnosis. It is found that the difference in each index between groups before and after training is significant (*P* < 0.05).  Figure 5(b) is the results of the main diagnosis selection errors of the neurosurgery department. There are 180 errors in the discharge case statistics before the training and 50 errors after the training. The statistics on the five types of main diagnosis selection errors are conducted, including that the main diagnosis is head trauma, tumor morphological code is not written, the rehabilitation Z code is not used, coding of disease sites is inaccurate, and the cause of injury poisoning is not written. It is found that the difference in each index between groups before and after training is significant (*P* < 0.05).

### 3.6. Results of Disease-Coding Errors of Cardiovascular Medicine, Burns Surgery, and Ophthalmology Departments

Results of disease-coding errors of cardiovascular medicine, burns surgery, and ophthalmology departments are shown in Figure 6.  Figure 6(a) is the results of the coding errors of the cardiovascular medicine department. There are 420 errors in the discharge case statistics before the training and 180 errors after the training. The statistics on the five types of disease-coding errors are conducted, including arrhythmia, myocardial infarction (MI), coronary heart disease (CHD), sudden coronary death (SCD), and myocardial ischemia. It is found that the difference in each index between groups before and after training is significant (*P* < 0.05).  Figure 6(b) is the result of disease-coding errors of the burns surgery department. There are 170 errors in the discharge case statistics before the training and 35 errors after the training. The statistics on the seven types of disease-coding errors are conducted, including that multiple burns are the main diagnosis, the burn degree and area not written, the burn site is not filled in accurately, scald/burn is not written clearly, coding of chilblain and frostbite is confusing, burn complications are coded, and the cause of injury poisoning is not coded. It is found that the difference in each index between groups before and after training is significant (*P* < 0.05).  Figure 6(c) is the results of disease-coding errors of the ophthalmology department. There are 160 errors in the discharge case statistics before the training and 30 errors after the training. The statistics on the five types of disease-coding errors are conducted, including that the diagnosis of the disease is filled incompletely, the disease diagnosis name localization is not accurate, coding choices are too general, the diagnosis name is not detailed, and the disease is not coded according to coding principles. It is found that the difference in each index between groups before and after training is significant (*P* < 0.05).

### 3.7. Automatic Annotation Results of the Medical Record Language

The results of automatic annotation of the medical record language under different artificial intelligence algorithms are statistically analyzed (Figure 7).

Figure 7 indicates that the accuracy rate, symptom precision, and symptom recall of BIRNN are higher than those of CNN and RNN, which indicates that BIRNN has better automatic annotation effect of pathological language.

## 4. Discussion

In medicine, disease classification reflects the medical level of a hospital to a certain extent. Disease classification refers to the scientific classification of various diseases through coding to provide a basis for clinical diagnosis and treatment. Hospital requirements for accurate classification of diseases have also increased the requirements for disease coders [13, 14]. EMR is defined in *The Basic Framework and Data Standard Electronic Medical Record of Electronic Medical Record* issued by the Ministry of Health as follows: an electronic medical record is a digital medical service record of clinical diagnosis and treatment, guidance, and intervention of outpatients and inpatients (or health care objects) by medical institutions. Studies have shown that coders need to collect, classify, organize, analyze, and use medical record information through the criteria for disease classification. It requires coders to fully understand the clinical knowledge of various diseases [15–17]. This experiment analyzes the reasons for the main diagnosis selection error. The coders are not familiar with the basic rules of the main diagnosis selection, which leads to the misunderstanding of the main diagnosis as an outpatient diagnosis. The classification of disease codes is unclear, and it is believed that the same names have the same codes. The result is the same as that of Nhut Pham et al. [18]. It is difficult to make accurate main diagnosis selection for situations with multiple diseases at the same time. Complications are not the main diagnosis. The morphological coding is mistaken as the main diagnosis. Some studies have found that some coders do not code according to specific medical purposes [19]. The classification of the treatment period and the recovery period is unclear. The disease is not coded according to the main diagnosis principles. It is wrong to regard some damage causes as the main diagnosis. Other investigations have found that when multiple fractures occur, some coders will mistake a certain fracture as the main diagnosis, causing errors [20]. When there is a complication, the previous disease is mistaken as the main diagnosis. The most serious injury is not taken as the main diagnosis. Rehabilitation treatment is not taken as the main diagnosis. The coding of many kinds of diseases is not detailed and accurate.

The experiment analyzes the causes of disease-coding errors. There is no merge coding for diseases that should be merged. Studies have found that coding undiagnosed diseases according to diagnosed diseases is also one of the reasons for coding errors [21]. When accompanied by complications, accurate coding is not performed. Patients of different ages are not coded differently. Drug-induced diseases are not coded correctly. The diseases are not coded according to different conditions. This is consistent with the results of Mahajan et al. [22]. The diseases are not coded according to different sites and different onset times. The diseases are not coded according to the specific classification and according to cause. When coding, it is not carried out in the order of first determining the site and then looking at the severity of the disease. Postoperative complication codes are inaccurate. The coding is not performed according to diagnostic purposes. The filling of the disease diagnosis is incomplete. The name of the disease diagnosis site is inaccurate. Coding selection is too general. The solutions to these problems are as follows. The relevant knowledge training is provided for coders and clinicians. The doctors are regulated to fill in medical record templates. The communication is enhanced between coders and medical staff. The new coding requirements should be mastered at any time. Tanno et al. [23] reviewed the history of changes in the classification and coding of allergic reactions and found that better ICD codes could reduce the mortality of allergic diseases.

This experiment shows that the main reason for the main diagnosis selection errors and coding errors for coders is that they do not fully understand the various diseases and their classification. Therefore, relevant training in this area should be strengthened.

## 5. Conclusion

The study analyzes the reasons for the wrong selection of main diagnosis before and after training in obstetrics and gynecology, endocrinology, oncology, orthopedics, and neurosurgery, as well as the wrong disease coding in these departments. It is found that the statistical errors of various diseases before and after training are significantly different between the groups. It shows that the coding personnel do not have a thorough understanding of various diseases and their specific classification, and the medical staff cannot clearly fill in the medical records of diseases. Therefore, the relevant training of coders and medical personnel should be strengthened. However, there are also some shortcomings, such as the small number of samples. Later, the scope of sample collection can be expanded to provide some support for the main diagnosis selection and disease-coding research.

## Figures and Tables

**Figure 1:** CT and ultrasound images. (a) The chest CT image of COVID-19 cases. (b) The segmented image of the pneumonia-infected area. (c) CT of the abdomen. (d) Ultrasound of the abdomen.

**Figure 2:** (a) Main diagnosis selection errors and (b) disease-coding errors of the obstetrics and gynecology department (^*∗*^*P* < 0.05).

**Figure 3:** (a) Main diagnosis selection errors and (b) disease-coding errors of the endocrinology department (^*∗*^*P* < 0.05).

**Figure 4:** (a) Main diagnosis selection errors and (b) disease-coding errors of orthopedics department (^*∗*^*P* < 0.05).

**Figure 5:** Main diagnosis selection errors of (a) oncology and (b) neurosurgery (^*∗*^*P* < 0.05).

**Figure 6:** Disease-coding errors of (a) cardiovascular medicine, (b) burns surgery, and (c) ophthalmology departments (^*∗*^*P* < 0.05).

**Figure 7:** Performance comparison of different artificial intelligence algorithms.

**Table 1:** Content of database construction of the embedded medical record knowledge system.

Descriptive knowledge of disease	Terms of disease characteristics and selection of entry
Conclusive knowledge of disease	Keywords given for pathological conclusion are given
Normative data content	Age
XML document input information	Restrictions on character entry

## Data Availability

The data used to support the findings of this study are available from the corresponding author upon request.
